# Effect of Huaiqihuang Granules Combined with Comprehensive Nursing on Children with Primary Nephrotic Syndrome

**DOI:** 10.1155/2022/3279503

**Published:** 2022-01-15

**Authors:** Guiyun Yang, Huanqin Yang, Shifang Cui, Jinling Shan

**Affiliations:** ^1^Child Health Care Department, Zhangqiu Maternity and Child Care Hospital, Jinan 250200, China; ^2^Department of Paediatrics, Zhangqiu Maternity and Child Care Hospital, Jinan 250200, China

## Abstract

**Background:**

To observe the effect of Huaiqihuang granules combined with comprehensive nursing intervention on children with primary nephrotic syndrome (PNS) and its effect on renal function index.

**Methods:**

A total of 104 patients were included, and the patients were randomly divided into two groups, with 52 cases in each group. The control group was treated with glucocorticoid, and the study group was treated with Huaiqihuang granules. The clinical efficacy of the two groups was observed. The levels of TG, TC, EGFR, 24 h UTP, BUN, Scr, IgA, IgG, IgM, IFN-*γ* and TNF-*α* were compared between two groups before and after treatment. The incidence of adverse reactions and recurrence rate after treatment were compared between the two groups.

**Results:**

The effective rate of the study group (94.23%) was significantly higher than that of the control group (78.85%). Before treatment, there was no significant difference in TG and TC levels between the two groups. After treatment, the levels of TG and TC in both groups were decreased, and the decrease was more obvious in the study group. Compared with before treatment, the levels of 24 h UTP, BUN, Scr, IFN-*γ*, and TNF-*α* in both groups were significantly decreased after treatment, while EGFR, IgA, IgG, and IgM levels were significantly increased. Compared with the control group, the changes of each index in the study group were more obvious after treatment. After treatment, the incidence of adverse reactions and recurrence rate in the study group were significantly lower than those in the control group.

**Conclusions:**

Huaiqihuang granules combined with comprehensive nursing treatment in children with PNS can reduce the occurrence of recent recurrence and adverse reactions and improve the cellular immune function and renal function.

## 1. Introduction

Nephrotic syndrome (NS) is a common glomerular disease in children. According to reports [1], 21% of children with NS are preschool children, especially at the age of 3–5, and the incidence is generally higher in boys than in girls. The occurrence of NS is related to immune dysfunction, abnormal structure of glomerular capillary wall, and genetic factors. NS is characterized by “three high and one low,” namely, massive proteinuria, hypoproteinemia, high edema, and hyperlipidemia. Primary nephrotic syndrome (PNS) accounts for about 90% of NS [2]. The most common clinical symptoms of PNS is edema, which occurs initially in the eyelids and then spread throughout the body, with decreased urine production. In severe cases, abdominal cavity or pleural effusion, hematuria, or even anuria may occur, which seriously affects the life and health of children [3]. Western medicine often use glucocorticoid treatment, which can control the development of the disease to a certain extent, but easy to relapse. Long-term application will produce more adverse reactions [4, 5], which seriously affect the body quality and life quality of children and increases the family burden. Traditional Chinese medicine (TCM) has a long history in the treatment of kidney diseases, and its therapeutic effect is worthy of affirmation. From the perspective of TCM, PNS is classified into “edema” and “asthenia,” and it is believed that the occurrence of PNS is caused by spleen deficiency and kidney deficiency. Huaiqihuang granules has the effect of nourishing Qi and Yin and can reduce proteinuria and protect renal function with its adjuvant treatment of PNS, which has synergistic effect with hormone and immunosuppression [6]. In addition, due to the younger age of children, there will inevitably be mood fluctuations in the treatment process, affecting the treatment effect. Nursing intervention is an important auxiliary measure for clinical treatment, which can improve the psychological status of children and the compliance of their families, improve the therapeutic effect, and reduce the occurrence of clinical complications [7, 8]. To demonstrate the above views, this study compared the therapeutic effects of Huaiqihuang granules in the treatment of children with PNS.

## 2. Materials and Methods

### 2.1. General Information

A total of 104 children with PNS hospitalized in Zhangqiu Maternity and Child Care Hospital from October 2017 to February 2020 were selected. There were 61 males and 43 females. The age ranged from 3 to 12 years old, with an average of 7.38 ± 3.45 years old. The course of disease ranged from 3 to 10 months, with an average of 6.67 ± 2.23 months. According to the random number table method, they were divided into study group and control group. This study was approved by the ethics Committee of Zhangqiu Maternity and Child Care Hospital. The patients of PNS children agreed to all treatment plans and signed the informed consent. There was no significant difference in gender, age, and course of disease between the two groups (Table 1).

### 2.2. Treatment Methods

The control group was treated with prednisolone tablets (Shanghai Shangyao Xinyi Pharmaceutical Co., Ltd., approval number: H31020771), 5 mg/time, 2-3 times/day. The study group was treated with prednisolone tablets and Huaiqihuang granules (Qidong Gaitianli Pharmaceutical Co., Ltd., approval number: B20020074), 10 g/time, 2 times/day. Both groups were treated for 3 months and followed up for 6 months after discharge.

### 2.3. Comprehensive Nursing Methods

Both groups were given consistent care during hospitalization. The details are as follows: (1) explain the basic knowledge and precautions of PNS to the children and their families, so that the children and their families can have more understanding of the treatment plan. The vital signs and adverse reactions of the children during treatment were closely monitored, and abnormal cases were handled in time. Do a good job of ward environmental care, daily ward cleaning and disinfection of the ward, and open the window for ventilation to keep the air clean. (2) Nursing staff should closely observe the psychological status of the children, timely guiding the negative emotions of the children, such as resistance and anxiety, and improve their treatment compliance. (3) In the diet, children should take in enough calories and control the intake of sodium salt. Calculate the protein content in food, ensure protein supply and give high-quality protein diet, such as lean meat, eggs, beef, chicken, duck meat, fish, and other types. Children with edema and oliguria should be given adequate vitamins. (4) If the children were accompanied by severe edema, it is necessary to strengthen the skin cleaning of the children. For bedridden children, we should help them to turn over many times, every 2 to 3 hours to turn over once, turn over action should ensure gentle, avoid chafing skin. Provide breathable and soft water cushion bed and keep the sheets clean and tidy.

### 2.4. Observation Indicators

Clinical efficacy was compared between the two groups. Significant effect [10]: the liver and kidney functions of the children returned to normal after treatment, and urinary protein was identified as negative. Effective: the quantification of 24 h urinary protein quantification (24 h UTP) decreased by 50% or more than before treatment, and renal function was stable. Ineffective: the 24 h UTP after treatment decreased by less than 50% compared with that before treatment. Total effective rate = (number of effective cases + number of effective cases)/total number of cases × 100%.

The levels of total cholesterol (TC), triglyceride (TG), 24 h UTP, estimated glomerular filtration rate (EGFR), serum creatinine (Scr) and blood urea nitrogen (BUN) were compared between the two groups before and after treatment. 6 mL early morning fasting venous blood was collected, centrifuged at 3000 r/min for 5 min, and the serum was separated and stored in a −20°C refrigerator. The serum detection was detected by ELISA (Shanghai Jianglai Biotechnology Co., Ltd.) in strict accordance with the kit instructions. 24 h urine samples were collected from the children, and after being stirred evenly, the 24 h UTP was detected and calculated.

The changes of immunoglobulin (IgG, IgA, and IgM) contents in the two groups were observed before and after treatment. The contents of IgG, IgA, and IgM were detected by the turbidimetric method (Shanghai Tongwei Co., Ltd.) strictly in accordance with the kit instructions.

Serum levels of tumor necrosis factor (TNF) and interferon *γ* (IFN-*γ*) were compared before and after treatment. The levels of TNF and IFN-*γ* were detected by ELISA method (Shanghai Yubo Biotechnology Co., LTD.) strictly in accordance with the kit instructions.

The incidence of adverse reactions during treatment and recurrence after treatment were compared between the two groups. Adverse reactions include leukopenia, thrombocytopenia, abnormal liver function, gastrointestinal discomfort, and elevated blood glucose. The recurrence rate of the two groups was observed after 6 months of follow-up. The determination criteria for recurrence [11]: after complete cure, the morning urine protein changed from negative to +++ or ++++ or the 24 h UTP ≥50 mg/kg or urine protein/creatinine (mg/mg) ≥2.0 for 3 consecutive days.

### 2.5. Statistical Analysis

SPSS22.0 was used for data analysis. The measurement data were represented by mean ± standard deviation. The counting data were represented by N (%), and comparison between groups was performed by *χ*^2^ test. *P* < 0.05 was considered statistically significant.

## 3. Results

### 3.1. Comparison of Clinical Efficacy between the Two Groups

The number of effective cases in the study group was 49, and the total effective rate was 94.23%. In the control group, 41 cases were treated effectively, and the total effective rate was 78.85% (Table 1).

### 3.2. Serum Lipid Levels Were Compared between the Two Groups before and after Treatment

Before treatment, there was no significant difference in TG and TC levels between the two groups (*P* < 0.05). After 30, 60, and 90 days of treatment, the levels of TG and TC in both groups decreased, and the decrease was more obvious in the study group (*P* < 0.05, Figure 1).

### 3.3. Comparison of Renal Function Level between the Two Groups before and after Treatment

Before treatment, there were no significant differences in EGFR, 24 h UTP, BUN, and Scr levels between the two groups (*P* > 0.05). Compared with before treatment, the levels of 24 h UTP, BUN, and Scr in both groups decreased significantly (*P* < 0.05), and EGFR levels were obviously increased (*P* < 0.05). Compared with the control group, the changes of each index level in the study group were more obvious after treatment (*P* < 0.05, Figure 2).

### 3.4. Comparison of Immunoglobulin between the Two Groups before and after Treatment

Before treatment, there were no significant differences in IgA, IgG, and IgM levels between the two groups (*P* > 0.05). Compared with before treatment, IgA, IgG, and IgM levels increased in both groups and more notably in the study group (*P* < 0.05, Figure 3).

### 3.5. The Incidence of Adverse Reactions and Recurrence Rate Were Compared between the Two Groups

After treatment, the incidence of adverse reactions was 9.62% in the study group and 32.69% in the control group (*P* < 0.05, Table 2). After treatment, the recurrence rate was 7.69% in the study group and 21.15% in the control group (*P* < 0.05, Table 3).

### 3.6. Serum Cytokine Levels Were Compared between the Two Groups before and after Treatment

Before treatment, there was no significant difference in serum IFN-*γ* and TNF-*α* levels between the two groups (*P* > 0.05). Compared with before treatment, serum IFN-*γ* and TNF-*α* levels in both groups decreased after treatment, and the decrease was more obvious in the study group (*P* < 0.05, Figure 4).

## 4. Discussion

PNS in children is a common kidney disease in pediatrics, and its common inducing factors include heredity, allergic reaction and immune dysfunction [12]. If not effectively restricted, long-term development will cause glomerular function and structure disorders, hinder the growth and development of children. Clinically, hormone therapy is often used for PNS, which has anti-inflammatory and immunosuppressive effects [13, 14]. Glucocorticoids are the first-line drugs in the treatment of PNS in modern medicine and are widely used in clinic, such as prednisolone tablets. Long-term use will lead to excessive dependence or drug resistance in children, and the therapeutic effect is still not ideal [15]. However, the biggest problem is that children are prone to PNS recurrence, which will bring more difficulties to the treatment. According to clinical experience and relevant reports [16–18], the most common cause of PNS recurrence is infection. The recurrence of kidney disease induced by infection accounts for more than 50%, and the recurrence caused by respiratory tract infection is the most common. Therefore, infection control is the primary prevention and treatment measure to prevent recurrence.

PNS belongs to the category of “edema” and “consumptive” in TCM, and its occurrence is caused by deficiency of lung, spleen, and kidney [6]. Huaiqihuang granules are composed of Huaier fungus, Lycii Fructus, and Polygonati Rhizoma, and have the effect of nourishing Qi and nourishing Yin. Combined with the comprehensive nursing methods, the treatment effect can be optimally improved and the immune system of the children can be significantly improved. The results of this study showed that the incidence and recurrence of adverse reactions in the study group were lower than those in the control group, indicating that Huaiqihuang granules combined with comprehensive care can reduce the incidence of respiratory infections and various adverse reactions and further control the recurrence of PNS. It has been reported [19, 20] that Huaiqihuang granules can also reduce nephrotic proteinuria and relieve nephropathy in children. The results of this study showed that the levels of 24 h UTP, BUN, and Scr in both groups were significantly decreased after treatment, EGFR levels were significantly increased. Compared with the control group, the changes of each index in the study group were more obvious after treatment. The results of our study were consistent with the above reports. The serum immunoglobulins IgG, IgA, and IgM in the study group were significantly higher than those in the control group, and the total effective rate in the study group was higher than that in the control group. The results showed that Huaiqihuang granules combined with comprehensive nursing had a better therapeutic effect on children with PNS. Huaiqihuang granules can play an immunomodulatory role among which Huaier focuses on supplementing Qi, Lycii Fructus focuses on nourishing Yin, and Polygonati Rhizoma has the effect of supplementing Qi and Yin [21]. The combination of the three herbs can not only nourish the essence of viscera but also benefit the essence of the five viscera as a whole, so as to realize the overall tonic effect. Many studies have shown that cytokines are closely related to the pathogenesis of nephropathy [22–24]. In many nephropathy-related studies [25–27], the expression or concentration levels of serum IFN cytokines presented conflicting results. TNF levels were agreed to be significantly elevated. Our results showed that serum IFN-*γ* and TNF-*α* levels decreased in both groups after treatment compared with before treatment, and the decrease was more obvious in the study group. It showed that Huaiqihuang granules combined with comprehensive nursing can effectively restrict the proliferation of connective tissue and reduce the permeability of cell membrane and capillary wall, so that inflammatory reaction can be alleviated. Children with PNS are often accompanied by metabolic disorders, which increase the synthesis of lipoprotein to hyperlipidemia, resulting in a large amount of cholesterol deposition in the intima of the artery, greatly increasing the risk of thrombosis and atherosclerosis [28]. The results of this study showed that the levels of TG and TC in the study group decreased more significantly than those in the control group, indicating that Huaiqihuang granules combined with comprehensive nursing can reduce the levels of TC and TG by immunosuppression of lipid metabolism.

## 5. Conclusion

To sum up, Huaiqihuang granules combined with comprehensive nursing reduce the adverse reactions of drugs, but also adjust the balance of immune cells disorders, improve the immune function of the body, have a good protective effect on the body kidney, and can significantly improve the treatment effect of children with PNS [9].

## Figures and Tables

**Figure 1:** Comparison of blood lipid levels between the two groups before and after treatment. The comparison of (a) TG levels and (b) TC levels between the two groups at 30, 60, and 90 days before treatment.

**Figure 2:** Comparison of renal function levels between the two groups before and after treatment. The comparison of (a) EGFR levels, (b) 24 h UTP levels, (c) BUN levels, and (d) Scr levels between the two groups before and after treatment.

**Figure 3:** Comparison of immunoglobulins between the two groups before and after treatment. The comparison of (a) IgA levels, (b) IgG, and (c) IgM levels before treatment between the two groups.

**Figure 4:** Comparison of serum cytokines levels between the two groups before and after treatment. The comparison of (a) serum IFN-*γ* levels and (b) serum TNF-*α* levels between the two groups before and after treatment.

**Table 1:** Comparison of clinical efficacy between the two groups (*n* (%)).

Group	*n*	Special effect	Valid	Invalid	Total effective rate
Study group	52	23	26	3	49 (94.23)
Control group	52	14	27	11	41 (78.85)
*χ* ^2^					6.779
*P*					0.034

**Table 2:** Comparison of the incidence of adverse reactions between the two groups after treatment (*n* (%)).

Groups	*N*	Thrombocytopenia	Leukopenia	Abnormal liver function	Gastrointestinal discomfort	Hyperglycemia	The total incidence
Study group	52	1	1	0	1	2	5 (9.62)
Control group	52	3	6	0	3	5	17 (32.69)
*χ* ^2^							6.144
*P*							<0.05

**Table 3:** Comparison of recurrence rates between the two groups after treatment (*n* (%)).

Groups	*n*	Positive urinary protein	Relapse
Study group	52	8 (15.38)	4 (7.69)
Control group	52	23 (44.23)	11 (21.15)
*χ* ^2^		4.353	4.720
*P*		<0.05	<0.05

## Data Availability

Data to support the findings of this study are available on reasonable request from the corresponding author.

## References

[1] Iijima K., Sako M., Nozu K. (2017). Rituximab for nephrotic syndrome in children. *Clinical and Experimental Nephrology*.

[2] Wang F., Zhang Y., Mao J. (2017). Spectrum of mutations in Chinese children with steroid-resistant nephrotic syndrome. *Pediatric Nephrology*.

[3] Hao S., Wu Y., Kang Y., Niu X., Zhu G., Huang W. (2020). A single-center analysis of primary nephrotic syndrome with acute pancreatitis in children. *Medicine*.

[4] Trautmann A., Vivarelli M., Vivarelli M. (2020). IPNA clinical practice recommendations for the diagnosis and management of children with steroid-resistant nephrotic syndrome. *Pediatric Nephrology*.

[5] Waller A. P., Agrawal S., Wolfgang K. J. (2020). Nephrotic syndrome‐associated hypercoagulopathy is alleviated by both pioglitazone and glucocorticoid which target two different nuclear receptors. *Physiological Reports*.

[6] Zhang X., Cheng Y., Zhou Q. (2020). The effect of Chinese traditional medicine huaiqihuang (HQH) on the protection of nephropathy. *Oxidative Medicine and Cellular Longevity*.

[7] Li F. X., Hou Y. L., Zhou L. S., Dong Y., Zhao J. W., Li Z. X. (2021). The status and model of children primary nephrotic syndrome in continuing nursing. *Annals of Palliative Medicine*.

[8] Yu X., Han C.-Y. (2021). Effect assessment of evidence-based nursing in combination with clinical nursing pathway on nephrotic syndrome care in children. *Medicine*.

[9] Pasini A., Benetti E., Conti G. (2017). The Italian Society for Pediatric Nephrology (SINePe) consensus document on the management of nephrotic syndrome in children: Part I - diagnosis and treatment of the first episode and the first relapse. *Italian Journal of Pediatrics*.

[10] Tiwari S., Seth A. (2016). Nephrotic syndrome in children - a tale of 50 years. *Indian Pediatrics*.

[11] Morello W., Puvinathan S., Puccio G. (2020). Post-transplant recurrence of steroid resistant nephrotic syndrome in children: the Italian experience. *Journal of Nephrology*.

[12] Moorani K. N., Hotchandani H. M., Zubair A. M., Lohana N. C., Veerwani N. R. (2019). Immunosuppressive therapy in children with primary nephrotic syndrome: single center experience, Karachi, Pakistan. *BMC Nephrology*.

[13] Che R., Zhang A. (2013). Mechanisms of glucocorticoid resistance in idiopathic nephrotic syndrome. *Kidney & Blood Pressure Research*.

[14] Zhao Y., Su B. G., Xiao H. J. (2017). Clinical characteristics of glucocorticoid-induced eye adverse reactions in children with primary nephrotic syndrome. *Beijing Da Xue Xue Bao Yi Xue Ban*.

[15] Lucafò M., Granata S., Bonten E. J. (2021). Hypomethylation of NLRP3 gene promoter discriminates glucocorticoid-resistant from glucocorticoid-sensitive idiopathic nephrotic syndrome patients. *Clinical and translational science*.

[16] Fine R. N. (2007). Recurrence of nephrotic syndrome/focal segmental glomerulosclerosis following renal transplantation in children. *Pediatric Nephrology*.

[17] Saeed B., Mazloum H. (2016). Recurrent nephrotic syndrome after renal transplant in children. *Experimental and Clinical Transplantation : Official Journal of the Middle East Society for Organ Transplantation*.

[18] Grenda R., Jarmużek W., Rubik J., Piątosa B., Prokurat S. (2016). Rituximab is not a “magic drug “ in post-transplant recurrence of nephrotic syndrome. *European Journal of Pediatrics*.

[19] Guo Y., Wang M., Mou J. (2018). Pretreatment of Huaiqihuang extractum protects against cisplatin-induced nephrotoxicity. *Scientific Reports*.

[20] Liu J., Yan H., Chen X. G., Mu Y. P. (2017). Effects of Huaiqihuang granules on immune function in children with severe Mycoplasma pneumoniae pneumonia. *Zhong Guo Dang Dai Er Ke Za Zhi*.

[21] Li T., Mao J., Huang L. (2016). Huaiqihuang may protect from proteinuria by resisting MPC5 podocyte damage via targeting p-ERK/CHOP pathway. *Bosnian Journal of Basic Medical Sciences*.

[22] Neuhaus T. J., Wadhwa M., Callard R., Barratt T. M. (1995). Increased IL-2, IL-4 and interferon-gamma (IFN-gamma) in steroid-sensitive nephrotic syndrome. *Clinical and Experimental Immunology*.

[23] Jafar T., Agrawal S., Mahdi A. A., Sharma R. K., Awasthi S., Agarwal G. G. (2011). Cytokine gene polymorphism in idiopathic nephrotic syndrome children. *Indian Journal of Clinical Biochemistry*.

[24] Carlotti A. P., Franco P. B., Elias L. L. (2004). Glucocorticoid receptors, in vitro steroid sensitivity, and cytokine secretion in idiopathic nephrotic syndrome. *Kidney International*.

[25] Agrawal S., Brier M. E., Kerlin B. A. (2021). Plasma cytokine profiling to predict steroid resistance in pediatric nephrotic syndrome. *Kidney International Reports*.

[26] Midan D. A. R., Elhelbawy N. G., Habib M. S. E., Ahmedy I. A., Noreldin R. I. (2017). Cytokine gene polymorphism in children with idiopathic nephrotic syndrome. *Iranian journal of kidney diseases*.

[27] Sadeghi-Bojd S., Hashemi M., Firoozi-Jahanigh M., Rezaei M., Sarani H., Taheri M. (2021). Lack of association between TNF-alpha rs1800629 (-308G > A) polymorphism and nephrotic syndrome. *Iran J Kidney Dis*.

[28] Zhang R. X., Zhang X., Zhang B. L., Liu Z. F., Lin S. X. (2021). Expression of adipokines in children with primary nephrotic syndrome and its association with hyperlipidemia. *Zhongguo dang dai er ke za zhi = Chinese journal of contemporary pediatrics*.

